# Bioprinting of Vascularized Tissue Scaffolds: Influence of Biopolymer, Cells, Growth Factors, and Gene Delivery

**DOI:** 10.1155/2019/9156921

**Published:** 2019-04-02

**Authors:** M. D. Sarker, Saman Naghieh, N. K. Sharma, Liqun Ning, Xiongbiao Chen

**Affiliations:** ^1^Division of Biomedical Engineering, College of Engineering, University of Saskatchewan, Saskatoon, SK, Canada; ^2^Department of Mechanical Engineering, College of Engineering, University of Saskatchewan, Saskatoon, SK, Canada

## Abstract

Over the past decades, tissue regeneration with scaffolds has achieved significant progress that would eventually be able to solve the worldwide crisis of tissue and organ regeneration. While the recent advancement in additive manufacturing technique has facilitated the biofabrication of scaffolds mimicking the host tissue, thick tissue regeneration remains challenging to date due to the growing complexity of interconnected, stable, and functional vascular network within the scaffold. Since the biological performance of scaffolds affects the blood vessel regeneration process, perfect selection and manipulation of biological factors (i.e., biopolymers, cells, growth factors, and gene delivery) are required to grow capillary and macro blood vessels. Therefore, in this study, a brief review has been presented regarding the recent progress in vasculature formation using single, dual, or multiple biological factors. Besides, a number of ways have been presented to incorporate these factors into scaffolds. The merits and shortcomings associated with the application of each factor have been highlighted, and future research direction has been suggested.

## 1. Introduction

Growing tissue in 3D scaffold requires functional and stable vascular network in order to maintain the viability and biological function of a large cell population. In recent years, unprecedented progress in additive manufacturing (AM) technique (i.e., extrusion and laser) has made possible the fabrication of complex vascular tree analogous to native tissue inside a scaffold [1]. While the AM technique provides the appropriate biophysical, structural, or topographical cues to the growing blood vessels, the precise selection and manipulation of scaffolding biopolymer, vascular cells, growth factors (GFs), and gene delivery approach significantly affect the formation of mature, stable, and functional vascular network in the tissue scaffolds [2, 3].

During blood vessel formation in the scaffolds, the interactions between biopolymer and vascular cells regulate the viability, proliferation, differentiation, and migration of incorporated cell populations [4]. As biopolymers are the primary building block of scaffolds, the selection of ideal or smart biopolymer affects the development of functional vasculature. Smart scaffolding biopolymer should be biocompatible, mechanically stable, biodegradable, non-toxic, and similar to specific ECM proteins. In addition, the selection of biopolymer depends on the anatomical territory where the scaffolds would be implanted and the chosen 3D fabrication approach. To date, different studies have explored a wide variety of synthetic, natural, and hybrid biopolymers to fabricate vascularized scaffold with conventional and AM technique [1]. However, only a few of them were able to synthesize polymers close to smart scaffolding biopolymer. Therefore, current research efforts are giving priority to synthesize ECM-like biopolymers that are bioprintable and biodegradable.

Vascular cells play a vital role in vasculature formation through proliferation, differentiation, and ECM protein generation. Particularly, in an ischemic tissue, endothelial cells (ECs) form capillary-like blood vessels through angiogenesis and vasculogenesis mechanisms. In tissue engineering approach, generally, the two mechanisms are harnessed in order to develop a vascular network within the scaffolds [4]. Until now, a number of studies have used vascular cells (i.e., ECs, smooth muscle cells, and pericytes) to vascularize tissue-engineered scaffolds. The cells were either incorporated in the scaffolds during biofabrication or postseeded on the outer surface of the scaffolds after preparation. Since regeneration of vascular tree requires the incorporation of large autologous cells in the vascular channels, generally, autologous cells are collected, expanded, and harvested prior to inclusion. Unfortunately, vascular cells gathered from old or diseased patients demonstrate poor proliferative ability, while the cell expansion is essential to create sufficient cell density in the vascular network. To tackle the issue, possible applications of stem and progenitor cells in the vasculature formation have been investigated over the years. Moreover, the coculture of multiple cell types and the behavior of vascular cells with respect to different scaffolding biopolymer have been reported in the recent studies.

*In vivo*, upregulation of various GFs facilitates the formation and maturation of vascular network. The ischemic tissue released several GFs alone, simultaneously or sequentially for a prolonged period that allows the development of stable vascular network [2]. To mimic the *in vivo* mechanism, until now, several GFs loading and release approaches have been developed that are proved effective for capillary blood vessel formation within the scaffolds. Since the released GFs demonstrate instability, a good number of studies have used transfected cells or gene-loaded biopolymer to obtain a prolonged or regulated release of GFs [3]. However, the gene delivery method requires vectors that are not free from shortcomings, and until now, a good number of research works have investigated how to tackle the issue.

Functional vasculature formation with scaffolds demands the perfect selection and use of several factors (i.e., scaffolding biopolymer, vascular cells, GFs, and gene delivery approach). To this end, a literature review is required that would allow us to select and manipulate the factors in the right fashion to obtain the growth of stable vascular network in the engineered construct. However, a review study encompassing the influence of the factors on scaffold vascularization remains unexplored to date. Consequently, in this study, a brief review has been conducted to focus on the recent advances in the factors for tissue vascularization. Besides, several important issues, advantages, and disadvantages associated with scaffolding biopolymer, vascular cells, GFs, and gene delivery approaches have been summarized, and directions for future research have been included.

## 2. Additive Manufacturing of Vascularized Construct

Additive manufacturing (AM) technique, also known as rapid prototyping (RP), has been used widely to create complex capillary networks. This technique includes extrusion-based and laser-based techniques. Inkjet-based bioprinting is likely used for tissue engineering applications because it ensures a relatively high cell density incorporated into scaffolds in comparison with the post-cell-seeding method [1].

### 2.1. Inkjet-Based 3D Bioprinting

The secretion of many biomolecules by cells is advantageous in the tissue generation process. That is why many studies recommended incorporating cells in the scaffolds at a high density. Hydrogels are cell-friendly biomaterials used in the extrusion-based bioprinting to fabricate structure in a layer-by-layer fashion as per a computer-aided design (CAD) [5, 6]. Two known generations of extrusion-based bioprinting methods are thermal- and piezoelectric-based bioprinting. Using such techniques, cell-incorporated hydrogel scaffolds can be created in a crosslinking solution. Hydrogels used for scaffold creation have a relatively high gelation rate, and it facilitates printing with a high speed of nozzle movement. Inkjet printing enables the incorporation of different types of cells into scaffolds while depositing in a controlled fashion and according to CAD design. For example, cell-incorporated alginate (as a hydrogel) scaffolds have been reported numerously while calcium chloride has been used as a crosslinker (alginate has been the main matrix for scaffolds creation) [7–11]. According to these studies, vascular networks grew inside the printed scaffolds in the *in vitro* and *in vivo* culture. In another study, bovine aortic endothelial cells, human amniotic fluid-derived stem cells, and canine smooth muscle cells were incorporated into alginate-collagen scaffolds fabricated by a thermal inkjet printer. This study showed vascularized tissues after an *in vivo* study [12]. Human microvascular endothelial cells (HMVECs) and thrombin solution mixed with fibrinogen in another study demonstrated aligned vessel-like structures along with the proliferated HMVECs [13]. Nonetheless, inkjet bioprinting shows some disadvantages including nozzle clogging, impossibility of printing high viscous biomaterials, and cell damage in the biofabrication process [14].

### 2.2. Extrusion-Based 3D Bioprinting

Extrusion-based bioprinting is another type of bioprinting technique used widely for the creation of vascularized structures (Figure 1(a)). This technique can fabricate vascular networks with sacrificial inks and makes possible printing biopolymers with poor printability. Such sacrificial templates are chosen carefully to avoid the use of cytotoxic organic solvents in generating vascular pattern [15–20]. Quite often, ECs are postseeded on scaffolds created by extrusion-based technique, and ECs then form a monolayer and facilitate mass transfer and vascularization [21]. In a study, a 3D construct was generated by extruding carbohydrate glass filaments. This 3D structure was then filled with a cell-incorporated (primary rat hepatocytes and fibroblast cells) agarose polymer matrix, and the sacrificial materials were removed. In the next step, the vascular lumens including human umbilical vein endothelial cells (HUVECs) were perfused with blood *in vivo*. The results show that the 3D vascularized construct with channels influences albumin secretion and urea synthesis by primary hepatocytes [22]. Nonetheless, the disadvantages of using this technique (e.g., a relatively high temperature during extrusion and nonhomogenous distribution of different cell types) limit its application. To address the issue, another innovative technique has been evolved to print various types of cells layer by layer than printing different types of cells together. Coprinting of fibroblast-laden GelMA, fugitive ink, and human neonatal dermal fibroblast-loaded GelMA has been reported elsewhere [23]. In this study, more than 95% cell viability has been observed for injected HUVECs.

Coaxial nozzle printing, a novel type of extrusion-based bioprinting, can fabricate core/shell structures, as reported in numerous studies [1, 24]. As an example, in a study, a flow of CaCl_2_ was used in the core side of a core/shell nozzle; meanwhile, a hydrogel was extruded through the shell side of nozzle [25]. In this technique, significant factors influencing the final structure of a hollow structure include the viscosity and concentration of biomaterial, as well as, the amount and concentration of applied crosslinker. These structures created through coaxial nozzle printing can be used to encapsulate various cell types into hydrogels. By modulating the factors that affect coaxial nozzle printing, 3D hollow structures with different mechanical properties can be created [26]. Furthermore, not only cells have been seeded in such structures but also ECs have been incorporated in these hollow structures [27]. In one study, human bone marrow stromal cells (hBMSCs) seeded on hollow scaffolds made of alginate-poly(vinyl alcohol) (PVA) showed an acceptable attachment after 14 days of *in vitro* study [26]. Similarly, cartilage progenitor cells (CPCs) incorporated into sodium alginate-based core/shell strands showed progress in cell viability after 3 days of incubation [27].

Generally speaking, natural, synthetic, or hybrid biopolymers are often used for bioprinting. Due to reasons such as uncontrolled degradation, biocompatibility issues, poor printability, and poor mechanical/biological properties, a combination of natural and synthetic biomaterials is recommended in the bioprinting of the vascular construct.

### 2.3. Laser-Based 3D Bioprinting

Laser-based bioprinting has been reported in numerous studies to create 2D and 3D cell patterning [29] (Figure 1(b)). This technique can print cells without any nozzle clogging while maintaining a high resolution. Vascularized structures have been observed in 3D structures created by laser-based bioprinting technique in several studies. For instance, HUVECs and human mesenchymal stem cells (hMSCs) were printed using this technique to create a cardiac patch, and the graft was transplanted in the infarcted zone of rat hearts. The patch increased blood vessel formation and significantly improved the function of the infarcted hearts [30]. A pattern on HUVEC incorporated into Matrigel™ was reported elsewhere to form a self-assembled vascular structure in the *in vitro* study [31]. The disadvantages of laser-based bioprinting technique are relatively long fabrication time, and laser-induced cell damage and such deficiencies limit this technique.

One of the laser-based bioprinting techniques is stereolithography, which is a maskless method and uses photosensitive materials [32]. Digital light projection (DLP) and laser-based stereolithography are known as laser-based bioprinting techniques implemented to create complex structures as per CAD design created through computer tomographic (CT) or magnetic resonance imaging (MRI) information [33]. The DLP method gains advantage of using a digital mirror device with thousands of small mirrors moved according to a digital signal. Once these small mirrors are moved, the laser beam is focused on the photo-curable biomaterial and it is cured as per CAD design. In another study, DLP was used to crosslink methacrylate (GelMA) solution using an ultraviolet (UV) light source and reflective dynamic photomasks. HUVECs were seeded on GelMA structure, and they maintained their phenotype during a 4-day study period [34]. Also, HUVECs showed a cord-like pattern after 4 days of *in vitro* study in scaffolds fabricated by a DLP system [35]. Some disadvantages of the DLP technique that limit its application include high expenses, the fabrication complexity of large structures, and cytotoxicity of photocurable biomaterials.

Laser-based stereolithography (LS), a photomaskless method, is another type of laser-based bioprinting technique. The printing speed rate of this technique is slower than DLP, but it is still an appropriate method to create large vascularized structures [36]. The LS method works based on a computer-controlled ultraviolet laser beam and this beam creates a pattern as per CAD design on a photocrosslinkable biomaterial [37]. Vascularized structures with complicated features have been created using this technique. Scaffolds printed using this technique and postseeded with ECs showed enhanced cell viability. However, cells incorporated into photocrosslinkable biomaterial showed low cell viability owing to the damage caused by laser beam with short wavelengths. This issue has been addressed through using tri-photon laser systems though (accuracy in the order of micron or nano) [38]. Studies have shown that, for instance, granulosa cells seeded on an epoxy-based vascular tree printed with laser-based bioprinting technique promote considerable cell growth along with continuous cell-cell junctions [39].

## 3. Scaffold Fabrication Biomaterial

Scaffold is a temporary structure that can be implanted *in vivo* to promote and guide the formation of vascular network (Table 1). To fabricate such a scaffold, a biomaterial with appropriate property (biochemical, biophysical, and mechanical) is required. Particularly, biomaterial should have the property like ECM, as such implanted scaffold can interact with vascular cells and thus support the survival, proliferation, differentiation, and migration of vascular cells by activating numerous signaling pathways. Besides, biomaterial should have sufficient mechanical strength in preserving the scaffold structure *in vivo* since implanted scaffold often experiences different types of forces (such as compression, shear, torsion, and tensile) which are responsible for structural destruction. In addition, biomaterial should demonstrate biocompatibility and controlled biodegradability to avoid post-implantation rejection, inflammation, and complexity. Based on the source or preparation method, biomaterials can be classified as synthetic, natural, and hybrid (Figure 2).

### 3.1. Synthetic Polymer

Over the last few decades, a wide range of synthetic materials has been explored in scaffold fabrication for tissue vascularization. Many of them demonstrate various attractive engineering features, superb mechanical properties, biodegradability, biocompatibility, and nontoxicity. However, the absence of bioactive molecules in the molecular structure limits the application of synthetic biomaterial in tissue vascularization. To overcome the shortcomings of bioactive molecule, tailored or protein-adsorbed synthetic polymers have been used in scaffold fabrication to date.

Aliphatic polyesters, silicon, poly(phosphoesters), hydrogel-based polymers, and poly(acrylonitrile-co-methylacrylate (PAN-MA) have frequently been studied for vascularization. Polyglycolic acid (PGA) is a biodegradable polymer which degrades through hydrolysis upon implantation. Copolymerization with other polymers (such as poly-L-lactic acid (PLLA), polyhydroxyalkanoates (PHAs), and polyethylene glycol (PEG)) can be used to eliminate the uncontrolled degradation of PGA [40–42]. *In vitro* and *in vivo* studies demonstrate that PGA scaffold facilitates the formation of blood vessel-like structures and collagen deposition [43, 44]. Scaffold fabricated with PLA-derived material showed angiogenic potential in different studies. Porous PLLA/collagen scaffold containing human aortic SMCs accelerated the formation of a smooth inner layer *in vitro* [45], VEGF-encapsulated PLGA microspheres-enhanced local angiogenesis in the mice model [46]. Besides, efforts were made in different studies to form vasculature *in vivo* with composites and derivatives of polycaprolactone (PCL) to overcome the slow degradation of PCL. Implanted PCL/PLA vascular graft aligned ECs and regulated ECM generation *in vivo* [47] and caused no postoperative complications for seven months postoperatively when used as a pulmonary bypass graft [48]. Likewise, SMCs-incorporated poly(L-lactide-co-ɛ-caprolactone) (PLCL) resulted in equivalent proliferation and alignment of SMC and collagen deposition similar to native tissues after eight weeks of *in vitro* culture [49].

Various composites and derivatives of polyhydroxyalkanoates demonstrate a wide range of mechanical properties and degradation rates and have been explored in vasculature formation. Implanted PGA-PHA scaffold seeded with ovine carotid artery cells in lambs maintained cellular growth, collagen production, and mechanical strength of grown tissue similar to that of native vessels [50]. In some studies, biodegradable polymeric scaffolds were used to release growth factors. Hydrolysis of PLGA and poly(ester urethane) urea fabricated-scaffolds released the encapsulated VEGF and FGF-2, respectively, that supported angiogenesis [46, 51]. Expanded polytetrafluoroethylene (PTFE), polyethylene terephthalate (Dacron), and polyurethane are some of the nondegradable synthetic polymers that are well known for various tissue vascularization applications. In particular, dacron, expanded PTFE, and polyurethane were used in several studies to prepare aortic graft, femoropopliteal bypass grafts, and hemodialysis, respectively.

### 3.2. Natural Polymer

Protein-based and polysaccharidic polymers have been explored frequently in numerous studies to form vascular tissues. While natural polymer possesses essential biochemical, physical, and topographic cues for vasculature formation, poor mechanical stability, high processing cost, and rapid degradation limit their applications. A good number of studies fabricated scaffolds with cells/growth factors loaded pure or composite natural materials (e.g., fibronectin, fibrin, elastin, silk fibroin, matrigel, and collagen) and reported vascular tissue formation *in vitro* and *in vivo*. Collagen scaffolds incorporated with DNA-encoding VEGF promoted vasculature growth when implanted subcutaneously into mice [55]. Further, subcutaneously implanted collagen grafts loaded with fibrinogen gel in rats underwent angiogenic sprouting from the femoral vessels. More vascular network formation was reported in the collagen/fibrinogen scaffolds compared to fibrinogen ones. In addition, adipose-derived stem cell- (ASC-) seeded collagen scaffolds enhanced greater vascular volume than collagen scaffolds alone [56]. Besides fibronectin, an ECM protein demonstrated the ability of capillary formation in different studies. Implanted collagen I/fibronectin gel seeded with EC and mesenchymal cell into mice promoted well-perfused and stable vascular network formation [57], and fibronectin-coated collagen modules into immunodeficient mice improved human vascular EC viability and blood vessel development compared to uncoated collagen modules [58].

Fibrin, a fibrous protein, is a reaction product of thrombin on fibrinogen and has the ability to form vasculature. However, poor mechanical and degradation property of fibrin led researchers to use a composite of fibrin to fabricate vascular constructs. Fibrin matrix facilitated the formation of a vascular capillary network *in vitro* when human microvascular ECs were seeded into a fibrin composite (90% fibrin and 10% collagen) containing either bFGF/TNF-*α* or VEGF/TNF-*α* [59]. Subcutaneously implanted porous PEG hydrogels loaded with fibrin in a rodent model facilitated the development of higher vascular density compared to hydrogel alone [60]. Besides, elastin has been investigated for vasculature formation as 28–32% of major blood vessels are composed of elastin [61]. *In vitro* elastin-derived peptides were seen to influence the migration and proliferation of ECs and thus promoted vascular network formation [62]. *In vivo*, greater cell population and homogeneous vascular network formation were identified throughout the arteriovenous (AV) loops implanted subcutaneously in the rats thigh loaded with collagen-elastin scaffolds compared to collagen-glycosaminoglycan scaffolds [63]. Apart from ECM protein, silk fibroin was also identified as a potential protein in tissue vascularization. When endothelial and osteoblast cells were cultured on 3D silk fibroin nets, microcapillary-like structures were seen due to the self-assembled vascular tissue formation over 42 days [64]. Such predeveloped capillary network inside a 3D silk fibroin scaffold well anastomosed and perfused with the host vasculature after 14 days of implantation into an immunodeficient mice [65].

Different studies explored a number of polysaccharide polymers (such as alginate, chitosan, and hyaluronic acid) for vascular tissue engineering applications. Alginate hydrogel does not possess attachment sites for vascular cells in the molecular structure; however, they can maintain satisfactory cell viability being hydrated. Several studies enhanced biofunctionality of alginate with crosslinked peptides and incorporated angiogenic factors and adsorbed proteins [66–68]. It has been reported that manipulation of physical cues (e.g., pore geometry) within the hydrogel scaffold affects vasculature formation. *In vivo*, human embryonic stem cell cultured into alginate scaffolds having 90% porosity and variable pore sizes (∼50–200 mm) created void and tube-like structures [69]. Chitosan, a combination of glucosamine and *N*-acetyl glucosamine units, has been investigated in tissue vascularization due to antibacterial activity [70]. Implanted chitosan scaffolds prepared with the particle aggregation method in the rat muscle-pocket model for 12 weeks promoted the neovascularization [71]. Besides, it was reported that chitosan blended polymers have the ability to deliver growth factors in a controlled fashion. Subcutaneously implanted chitosan-4-hydroxylphenyl acetamide hydrogel loaded with human adipose-derived stromal cells (ADSC) and PDGF in nude female mice released cells and growth factor in a controlled manner that promoted vascularization [72]. Further, hyaluronic acid, an anionic and nonsulfated glycosaminoglycan, demonstrated reasonable successes in vasculature formation. For example, implanted spongy-like hydrogel (gellan gum-HA) into an ischemic hind limb of mice grew vascular network through a prolonged release of HA [73], and subcutaneously injected HA/recombinant gelatin hydrogel in the rats promoted vascular network developments over 4 weeks [74].

## 4. Selection and Addition of Cells

ECs, smooth muscle cells (SMCs), and pericytes are seen in the majority of the blood vessels *in vivo* [80]. These cells can be harvested from autologous, xenogenic, or allogenic sources [81]. However, the use of xenogenic or allogenic vascular cells provokes host immune response and thus promotes various complications. In contrast, autologous ECs, endothelial progenitor cells (EPCs), and stem cells incorporated vascular grafts implanted in the host body remain biocompatible for long period and does not undergo immunological rejection. ECs and SMCs harvested from various sources (e.g., umbilical vein, dermal microvessel, omentum fat, and carotid artery) were frequently investigated in angiogenesis and vasculogenesis studies [82, 83]. However, ECs harvested from different sources are dissimilar in morphology and functionality, and therefore, target specific ECs should be used in tissue vascularization to avoid complexities [84, 85]. Preliminary effort to promote vasculature with monoculture of cells had achieved some successes. Subcutaneously injected Matrigel/HUVEC suspension into mice formed mature blood vessels that remained functional till 100 days [86], implanted PLLA scaffolds loaded with human dermal microvascular endothelial cells (HDMECs) in the mice model grew functional microvessels that eventually got connected with the host vasculature [87], and calf pulmonary microvessel-derived ECs grew capillary-like networks under hypoxic condition within 3 days of *in vitro* culture [88].

*In vivo*, the interaction between cell-cell, cell-ECM, and cell-biochemical molecules regulate the formation of vasculature. Therefore, multiple cell-loaded grafts were used in different studies to promote vascular network (Figure 3). However, the appropriate cell types, ratio of incorporation, and functional manipulation have still remained unsolved. Coculture of ECs and pericytes on a prepatterned fibrin matrix formed capillaries with reduced diameter and permeability. In addition, such capillaries showed a greater number of junctions and branches compared to tubes formed by EC monoculture [89]. Since SMCs stabilize the blood vessels, ECs were cocultured with SMCs in a decellularized intestinal submucosa matrix in mice to obtain mature vascular tissue. The combination of cells promoted vascular network that was well perfused and integrated with host vascular bed 1 month postoperatively [90]. Similarly, coculture of microvascular ECs and human pulmonary artery-derived SMCs into a PLLA/Matrigel graft made the nascent blood vessel stable in immunocompromised mice. Moreover, the capillary bed anastomosed with the host vasculature within the 7 days of implantation [91]. Besides, another mural cell fibroblasts was investigated in tissue vascularization as implanted Matrigel plugs loaded with neonatal human dermal fibroblasts provoked capillary invasion from host vasculature [92]. The success of fibroblasts cell culture-motivated researcher to conduct the coculture of human dermal fibroblasts and HUVECs into microcarrier beads. The coculture of cells formed capillary-like sprouts within a fibrin-graft after 2–3 days and lumen containing capillaries after 8–14 days of *in vitro* culture [93]. Similarly, the formation of a capillary-like structure was reported in the cocultures of human osteoprogenitor cells/HUVECs [94], cardiomyocytes/HUVECs, [95], and osteoblasts/endothelial cells [96]. Taken all together, it can be concluded that cocultured ECs and tissue-specific or mural cells within an engineered construct have the capacity to promote vasculature in a macroscale and microscale range. However, some major shortcomings, such as inadequate availability, poor proliferation capability, prolonged time of proliferation, and poor functionality, limit the application of mature cells in vascular tissue engineering [97].

Time delay in vasculature formation inside a neotissue causes necrosis. Thus, most of the cell population undergoes apoptosis and tissue regeneration fails. In this regard, incorporation of stem cells into a vascular graft could be a reasonable solution as stem cells show rapid and high proliferation and superb differentiation ability to form vascular network [98]. MSCs obtained from various sources (bone marrow, adipose tissue, blood, and dermis) have the potential to differentiate into perivascular cells (e.g., SMCs) *in vivo*. Coculture of HUVECs and bone marrow-derived MSCs into collagen gel implanted in an immunodeficient mouse caused the differentiation of MSCs into perivascular cells. Moreover, the grown vascular bed within the graft stayed functional and stable beyond 130 days after implantation [99]. Besides, when MSC and peripheral blood-derived outgrowth endothelial cells (OECs) were cocultured in the medium containing either osteogenic differentiation medium (ODM) or endothelial cell growth medium (EGM), more microvessel-like stable structures were observed in the EGM compared to ODM after 2 weeks of *in vitro* culture. This study demonstrates the effect of specific culture media in vasculature formation [100]. Although many reasonable results were obtained using stem cells *in vitro* and *in vivo*, post-implantation complications (such as formation of atheromas, teratomas, tumors, and retinopathies), uncontrolled differentiation, and ethical issues are the major concerns related to stem cell applications that are still remained unsettled [98].

Progenitor cells are more convenient than stem cells in vascular tissue engineering. In different studies, EPCs showed greater commitment to EC differentiation compared to stem cells under the regulation of angiogenic factors, biomolecules, and shear stresses [104]. Originating from different sources (e.g., umbilical cord and peripheral blood, bone marrow, and liver tissue), EPCs demonstrated significant proliferative and angiogenic properties reported elsewhere [105]. Selection of right combinations of cells in coculture, scaffold design parameters, and culture media determines the success of microvessel formation with EPCs [106]. To grow macro blood vessel, decellularized porcine iliac vessels seeded with EPCs were implanted as a carotid graft in sheep. The recellularized vessels performed similar to native carotid arteries for 130 days postoperatively [107]. Besides, coculture of MSCs and EPCs in the 3D polyurethane (PU) scaffolds accelerated the formation of luminal tubular structures after 7 days of *in vitro* culture [108].

Perfusion bioreactors are quite effective in postfabrication cell seeding in a controlled and homogeneous fashion throughout the vascular graft. In a coculture system, the temporal and spatial protocol of cell seeding determines the success of vascularized tissue formation. For example, coseeding of ECs, fibroblasts, and cardiomyocytes in Matrigel formed cardiac tissue-like organoid structure where capillary network was seen absent [109]. To overcome the issue, sequential (24-hour time delay) seeding of ECs, fibroblasts, and cardiomyocytes in Matrigel was followed. This technique promoted tissue and capillary formation in the grafts [110]. However, such seeding approach requires porous scaffolds having microchannels and chemoattractant properties to enhance cell function [111].

## 5. Choice and Addition of Growth Factors

*In vivo*, angiogenic factors play a significant role in forming a vascular network through angiogenesis and vasculogenesis. Indeed, vasculature within tissue is formed through the combined influence of multiple angiogenic factors. In different studies, vascular endothelial growth factor (VEGF), platelet-derived growth factor (PDGF), fibroblast growth factor, angiopoietins (Ang), transforming growth factor-*β* (TGF-*β*), sphingosine-1-phosphate, and hepatocyte growth factor (HGF) have frequently been explored for tissue vascularization. Direct dosing in the biologic tissue reduces the bioactivity of GFs, whereas delivering through a biological graft ensures the safety and protection of GFs from harsh proteolytic milieu. Sequential, spatial and temporal delivery of growth factors (GF) from a vascular graft showed a significant effect on the capillary formation and vessel maturation in different studies. It was reported that early delivery of blood vessel stabilization factors deters ECs from sprouting, while delayed delivery of angiogenic factors degenerates the nascent blood vessels inhibiting the function of mural cells [112].

To vascularize an engineered graft, researchers have explored versatile approaches and techniques. Many studies used surface coating, encapsulation, impregnation, diffusion, and immersion technique to incorporate GFs in the vascular construct. While such GF-loaded grafts are cultured *in vivo* or *in vitro*, several factors, such as fabrication materials, GF incorporation method, and types of bonding (e.g., physical and covalent) between biopolymer and GF regulate the release pattern of the GFs (Figure 4). Researchers investigated a number of biopolymers including collagen, fibronectin, chondroitin sulfate, heparin sulfate, laminin, HA, and GF-specific peptides to immobilize GFs on the outer surface and internal structure of a vascular graft [113]. Apart from the physical attachment of GFs, covalently conjugated VEGF onto collagen scaffolds promoted the penetration, viability, and proliferation of ECs in the collagen scaffold compared to soluble VEGF [114].

To date, researchers have explored a number of strategies to load GFs in the engineered constructs. Among them, direct loading is the simplest one where GFs are mixed with biopolymer before gelation. Although such technique causes inefficient incorporation, uncontrolled release, and loss of bioactivity of GFs, several studies reported some successes of direct loading approach in forming capillaries [115]. When VEGF and Ang-1 loaded hyaluronan (HA) hydrogels were implanted in the ear pinnae of mice, a significantly higher microvessel density was observed in the treated groups than controls after 14 days of implantation [116]. Further, the sequential release of GFs was explored experimentally by manipulating the phase of GF incorporated biopolymers. When PDGF-loaded PLGA particles were incorporated into a VEGF mixed porous poly(lactide-co-glycolide) (PLG) scaffold, a sequential release of VEGF and PDGF was obtained. Such sequential delivery of VEGF and PDGF grew mature, dense, thick and large blood vessels [117].

For the sustained release of GFs, use of micro/nanocarriers is a better choice to incorporate GFs than the direct loading method [115]. Nondegradable carriers show an initial burst of GFs and were not suitable for sequential release of multiple GFs, whereas degradable carriers can release one or more GFs at a programmed rate over an extended period maintaining a certain concentration [118]. To evaluate GFs release pattern from microsphere, neonatal intestinal organoid units seeded on PGA scaffold containing VEGF-loaded PLGA microspheres were implanted in the omentum of recipient rats. Sustained release of VEGF upregulated better microvasculature formation than empty microsphere-treated groups after 4 weeks of implantation [119]. The success of microparticle in sustained release of GFs led researchers to explore the efficacy of nanoparticle in GF release. In a study, VEGF-loaded mesoporous silica nanoparticle was incorporated into a type I collagen sponge and then implanted in the chick chorioallantoic membrane (CAM) model. Such composite scaffold significantly increased the number of blood vessels compared to VEGF-free scaffold and released VEGF over 28 days *in vitro* [120]. Similarly, VEGF-incorporated nanoparticles (VEGF-NPs) implanted in a hindlimb ischemia model of rabbit promoted higher capillary density, a greater number of collateral arteries, and increased blood perfusion in VEGF-NP-treated limbs compared to VEGF- or nanoparticle-treated groups. In addition, a sustained release of VEGF for 28 days *in vivo* was reported [121].

Different combinations of growth factors demand different delivery approaches (e.g., simultaneous, sequential, and spatiotemporal) which has been reported as very effective in vasculature formation. For example, simultaneous release of VEGF and FGF-2 from collagen-heparin scaffolds in rats promoted more dense and mature blood vessels compared to the controls [122], and dual delivery of VEGF and Ang-1 from hyaluronan hydrogels in mice generated the best angiogenic response compared to controls 14 days postoperatively [116]. In contrast, sequential delivery of VEGF and S1P from Matrigel in mice grew more mature micro blood vessels than the sequential delivery of GFs in reverse order, single factor or dual factor delivery [112], and the successive release of VEGF and PDGF from PLGA scaffolds in mice significantly enhanced the size and maturity of blood vessels compared to controls 6 weeks after implantation [123]. Indeed, to form a stable vasculature, sustained and sequential release of multiple GFs is required from vascular graft. To address this issue, different studies coated the vascular construct or carriers with multiple layers of various degradation rates and found the approach quite effective in attaining controlled and sustained release of GFs. Besides, the successive layers prepared with various biopolymers capable of forming different types of bonds with GFs resulted in the desired release pattern of GFs over time. Instead of multiple biopolymers, single polymer having dissimilar affinities (affinity binding constants, *K*_A_) for GFs was investigated to prepare a coating layer that would release GFs in a sequential manner after implantation. GFs having higher *K*_A_ value for heparin or alginate sulfate was found to release slowly compared to GFs having lower *K*_A_ value. When such affinity-based alginate sulfate scaffolds containing VEGF, PDGF, and TGF-*β*1 were subcutaneously implanted in the rats, 3-fold higher percentage of mature blood vessels were seen than in the GF-adsorbed scaffolds 3 months postoperatively [124].

Since heparin shows an affinity for different angiogenic factors, covalently bound heparin with vascular construct was studied to bind GFs physically. In a study, covalently attached heparin sulfate (HS) with collagen was used to bind bFGF physically. When such scaffolds were subcutaneously implanted in rats, improved vascularization was observed throughout the construct compared to collagen-HS or collagen/bFGF grafts over 10 weeks after implantation [125]. Besides, recombinant proteins showed the ability in vasculature formation, while the proteins attach to specific binding sites of the ECM protein reported elsewhere. Since hepatocyte growth factor (HGF) shows short half-life, HGF was fused to a collagen-binding domain (CBD) to prepare CBD-HGF protein. When this recombinant protein was used in the injured carotid artery model in rats, CBD-HGF accelerated the re-endothelialization and neointimal formation compared with HGF-treated rats [126]. Similarly, CBD-HGF-bound collagen sponges implanted subcutaneously in rats increased the blood vessel count 4–6-fold greater compared to control 7 days postoperatively [127]. Tip cells of the vascular sprouts grow in the direction of gradient guidance cues [128]. Therefore, incorporation of the gradient of an angiogenic factor from the outer surface towards the inner core of a tissue scaffold is an effective strategy to grow vascular plexus throughout the neotissue. Since the excessive release of GFs causes leaky, immature, and unstable vascular bed, researchers investigated the cell-demanded release of GFs from a vascular construct in different studies [129]. Since ECs secret MMPs to degrade ECM in the capillary formation process *in vivo*, application of matrix metalloproteinases (MMPs)-degradable biopolymers in the vascular grafts facilitated the cell-demanded release of GFs in different studies [130]. Besides, platelet-rich plasma (PRP) was explored in different studies since they contain a naturally defined ratio of GFs useful in vasculature formation. In a study, when PRP-loaded gelatin hydrogels were implanted into the ischemic hindlimb of rats, a greater microvessel density was observed in the PRP-gel group compared to platelet-poor plasma or PRP groups 4 weeks postoperatively [131]. Although such plasma is available, inexpensive, and biocompatible, short half-lives of released GFs is one of the major shortcomings that need more investigations [132].

Apart from direct delivery strategy, researchers have also investigated a number of indirect delivery approaches to stimulate specific cells to release GFs on demand. Several studies showed that the regulation of antibiotics, electric fields, magnetic fields, light, and ultrasound triggers the GF release mechanism. For example, photodegradable PEG-based hydrogels released drugs in the presence of light [133], alginate ferrogels containing iron oxide nanoparticles released TGF-*β*1 in a sustained fashion under the influence of a magnetic field [134], platelet-rich plasma caused differential release of growth factors under pulsed electric fields [135], and antibiotic-sensing hydrogel at the addition of albamycin triggered the release of VEGF_121_ which promoted the proliferation of HUVECs [136]. Further, when ultrasound was applied to stimulate human mandibular peripheral blood monocytes, osteoblasts, and gingival fibroblasts, angiogenic factors (e.g., VEGF, IL-8, and bFGF) were obtained for both traditional and long wave frequencies [137].

## 6. Gene Therapy

The use of GFs in the engineered grafts results in stable and mature vascular network reported in different studies. However, short half-lives of the GFs need to be overcome to improve the efficiency of such an approach. To address this issue, a number of studies have used suitable vectors (e.g., viral and nonviral) to transfect specific cells in obtaining prolonged expression of target proteins [138] (Figure 5). In general, viral vectors offer higher cell transfection efficiency compared to nonviral one. Several viral vectors including retroviral, lentiviral, adenoviral, and adeno-associated viral vectors have frequently been explored to transfect tissue-specific cells. Both retroviral and lentiviral vectors demonstrate the size restriction of insertable genes and potential risk of mutagenesis [139]. Besides, adenoviral vectors show short-term transgene expression and high immune response, while adeno-associated viral vectors display long-term transgene expression and low immune response [140]. However, both vectors show the size constraint of insertable genes [141]. To avoid immunogenic and mutagenic complexity, researchers came up with alternative vectors called nonviral vectors. Such vectors are also cheap, nontoxic, applicable to any size of gene sequence, and ineffective in cell transfection [142]. In this regard, a number of studies explored physical and chemical methods to enhance transfection efficiency. Unfortunately, each method showed their own shortcomings; for example, while the physical approach caused significant cell damage, the chemical method resulted in cell cytotoxicity [143].

In several studies, genes were delivered to obtain sustained release of angiogenic factors from cells either by incorporating genetic vectors modified cells into the grafts or seeding cells on the scaffolds containing genetic vectors. Such approach ensures the release of growth factors for a long time and thus promotes vasculature formation. Besides, scaffold-based gene delivery technique is economic, gene protective from enzymatic degradation and slightly immunogenic to host tissue. A number of studies have explored micro/nanospheres, hydrogels, or electrospun constructs to deliver genetic vectors or modified cells. Hydrogels are potential biomaterials for incorporating genetic vectors since many hydrogels showed desired biodegradability, cell viability, and printability reported elsewhere [144]. When heparin-chitosan nanoparticle-functionalized PEG hydrogel was used to release lentiviral vector locally, overexpressed sonic hedgehog and VEGF promoted capillary vessel formation in the scaffold compared to either VEGF-delivering or control hydrogels [145]. The effect of pore size of the polyplex-loaded hydrogels on the transfection efficiency of infiltrating cells *in vivo* was investigated in a study. Subcutaneously implanted porous hyaluronic acid hydrogels loaded with pro-angiogenic (pVEGF) nanoparticles in mice caused more efficient cell transfection and vasculature formation than the nonporous one by 6 weeks [146]. To evaluate the angiogenic efficiency of other GF encoding plasmid rather than VEGF, FGF-4 plasmid-incorporated gelatin hydrogel (GHG) was injected into the hindlimb muscle of mice and rabbits. Gelatin hydrogel released gene over 28 days which promoted angiogenesis in the newly developed tissues in the GHG-FGF4 group than the naked FGF4-gene incorporated group four weeks after gene transfer [147]. Similarly, subcutaneously implanted PLG sponges loaded with plasmid-encoding PDGF improved ECM deposition and capillary formation in rats compared to the directly injected plasmid [148].

Injected plasmid-mediated VEGF gene loaded PLGA nanoparticles into ischemic myocardium tissue of rabbit caused a higher capillary number compared to the naked plasmid DNA (pDNA) group [149]. When VEGF plasmid incorporated PLGA nanospheres were injected into skeletal muscle of mice, more capillary blood vessels were seen within 4 weeks compared to injected naked pDNA or pDNA-loaded polyethylenimine (PEI) nanospheres [150]. Although promising, the localized delivery of nanoparticle in the tissue is difficult since they demonstrate a nonideal release profile [151]. Besides, cost-effective electrospun nanofibers containing a large surface-to-volume ratio, highly interconnected pores, and ECM-like structure significantly enhance tissue formation. Therefore, a number of studies have investigated the plasmid gene delivery from nanofilaments to promote vasculature. For example, electrospun poly(dl-lactide)–poly(ethylene glycol) (PELA) nanofibers loaded with calcium phosphate (CP) nanoparticles containing multiple plasmids (pVEGF and pbFGF) were seen to release plasmid genes over a sustained period (4 weeks) and showed significantly less cytotoxicity and inflammation reaction than PEI-pDNA nanoparticles after implantation *in vivo*. When such scaffolds (PELA/CP-pVEGF/CP-pbFGF) were subcutaneously implanted in rats, a significantly higher density of mature blood vessels was seen in the newly developed tissue than those containing individual plasmid [152]. PEI polyplexes containing pbFGF and pVEGF were incorporated into the PEG core of PELA fiber sheath prepared with the core-sheath electrospinning method. Such PELA/PEG nanofibers released pbFGF and pVEGF for a prolonged period (4 weeks) *in vitro* that promoted HUVECs attachment, viability, transfection, and secretion of ECM protein. When core-shell nanofibers were implanted subcutaneously in rats, significantly higher density of mature vessels was observed in the pbFGF- and pVEGF-encapsulated group compared to either pbFGF- or pVEGF-incorporated group [153]. However, drawbacks such as poor transfection efficiency and process-induced loss of bioactivity of incorporated plasmid genes limit the application of the electrospun method in gene delivery [154].

Although numerous studies reported stem cells as a promoter of vascularization, poor expression of secreted angiogenic factors and low cell viability are the major shortcomings of stem cells that need to be optimized. Instead of loading genetic vectors, a number of studies have used transfected stem cell-loaded scaffolds to promote vascularization. Such strategy improves the transfection efficiency of genetic vectors, viability of stem cells, and sustained release of angiogenic factors in the culture. Moreover, viral vector-associated immune rejection *in vivo* can be overcome by ex vivo transfection. For example, adenovirus encoding cDNA of VEGF was used to transfect the adipose-derived stromal cells (ADSCs). While PLGA microspheres seeded with ECs and transfected ADSCs were implanted on the dorsal region in mice, higher capillary density was observed in the scaffolds seeded with both ECs and transfected ADSCs compared to nontransfected ADSCs or EC-seeded microspheres [155]. Besides, researchers investigated the efficiency of genetic vectors in transfecting human-derived stem cells. In a study, nanoparticles composed of optimized poly(*β*-amino esters) (PBAE)-hVEGF were used to transfect hMSCs and human embryonic stem cell-derived cells (hESdCs). Such PBAE/VEGF gene transfected stem cells were transplanted in a hindlimb ischemia model in mice and 2- to 4-times higher capillary densities were found 2 weeks after implantation compared to controls or cells transfected with lipofectamine 2000/VEGF genes [156].

## 7. Summary and Future Research Directions

The success of tissue and organ regeneration largely depends on the formation of mature and well-perfused vascular network within the developing tissue. To date, a significant progress has been achieved in the printing of vascular construct. Since the scaffolding material has a profound effect on tissue growth, a good number of studies have been conducted to explore the appropriate biomaterial including natural and synthetic polymers. Interestingly, while natural biomaterial possesses cell-binding motifs and promotes cell-biomaterial interaction, poor mechanical stability limits their applications. In contrast, synthetic polymers show improved mechanical stability although they lack cell-binding sites. To handle these issues, hybrid or composite polymers were implemented in scaffold preparation. While implantation of acellular scaffolds facilitated tissue and vasculature formation to some extent, the invasion of the scar of fibrous tissue into the scaffolds remained problematical. Although migration of cells from host site was identified in the acellular scaffolds, tissue regeneration was unsatisfactory due to the random spatial settlements of the migrated cell population. The incorporation of tissue-specific or vascular cells in the scaffold solved the problem of cell positioning; however, this approach opens up other complexities. Several challenges have been experienced in the application of autologous, allogenic, and xenogenic vascular cells in the engineered construct described earlier. Stem cells have also been used instead of primary cells to eliminate the shortcomings, but the uncontrolled differentiation towards vascular cell lineage remains unsolved. In contrast, stem cells derived from fetal sources (e.g., placenta, umbilical cord, and amniotic fluid) are not tumorigenic and have the potential to grow vasculature. Also, the progenitor vascular cells have been found to be more devoted to specific cell lineage and promoter of capillary blood vessel formation compared to stem cells. Besides, in mature and stable capillary formation, the coculture of ECs and mural cells has been seen more effective compared to the monoculture system. Particularly, in a coculture system, the temporal and spatial techniques of cell seeding, cell ratio, and composition of culture media significantly regulate the vasculature formation. Since *in vivo* angiogenesis and vasculogenesis take place under the upregulation of multiple growth factors, GFs-loaded acellular and bioprinted scaffolds have been studied to promote capillary formation. A number of studies conclude that sequential and prolonged release of multiple GFs are the prerequisite for the formation of mature capillaries. Use of micro/nanocarriers, coatings, heparin sulfate, and covalent binding has made possible to deliver GFs in a controlled and prolonged fashion. Apart from sustained release, the release-on-demand approach can efficiently reduce the wastage of GFs from vascular graft. Even though GFs are effective in vasculature formation, short half-lives and high production cost of GFs led researchers to modify cells with genetic vectors. The viral vectors demonstrate higher gene transfection efficiency compared to nonviral one, however not free from immunogenic and mutagenic complexities. Transfection efficiency of viral vectors can be improved by incorporating ex vivo transfected cells into the scaffolds. The incorporated cells can maintain the overexpression of VEGF for a sustained period which is supportive in the formation of blood capillaries. To avoid the immunogenic and mutagenic complexity of viral vectors and increase the gene loading capacity, a good number of studies have synthesized and investigated nonviral vectors to date. However, the plasmid vectors have demonstrated poor cell transfection efficiency in different studies. To overcome the issue, several physical (electrotransfer, sonoporation, etc.) and chemical (lipoplexes, polyplexes, etc.) approaches have been explored and found convincing results in transfecting cell populations. Although a significant progress has been taken place in the past years, further research is needed in the area to overcome the transfection-associated complexities.

Tissue and organ regeneration requires smart biopolymer that would provide necessary physical and biochemical cues during tissue regeneration, as well as eventually gets replaced by the newly grown tissue. Unfortunately, neither natural nor synthetic polymer demonstrates all the desired properties. Therefore, research efforts should be continued to synthesize biocompatible and mechanically stable biopolymer with tailored biological property. Besides, more research is required to use nonimmunogenic and nontumorigenic fetal-derived stem cells for tissue vascularization. Since adeno-associated and nonviral vectors have the least risk of mutagenesis, future research should be conducted to harness these vectors in growth factors secretion for tissue engineering applications.

## Figures and Tables

**Figure 1:** Bioprinting with additive manufacturing technique: (a) extrusion-based vascularized scaffolds containing multilevel fluidic channels (reprinted with permission from [28] and (b) schematic of laser-based bioprinting technique (reprinted with permission from [1]).

**Figure 2:** Biomaterials and their effect on vascularization: (a) collagen scaffold (left), surface (middle), and cross section (right) and (b) harvested scaffolds at 1 and 4 weeks along with histological results ((a) and (b) reproduced with permission from [56]), (c) hydrogel swelling rate changes (upper row, scale bar: 2 mm) MSC encapsulation in 30, 50, and 80% DoF GelMA hydrogels (bottom row, scale bar: 200 *µ*m) (reproduced with permission from [75]), (d) SEM images of 5%, 10%, and 15% (w/v) GelMA hydrogels (left to right, reproduced with permission from [76]), (e) bioplotted 3% (w/v) alginate scaffold and SEM images, (f) control micrograph of expansive fibrin network (thrombin has been added to platelet-rich plasma, scale bar showing one micron, reproduced with permission from [77]), (g) SEM image of TA-PEG-gelatin hydrogel and the TA-PEG-gelatin/BCP hydrogel composite with 5% BCP amount (reproduced with permission from [78]), (h) SEM image of freeze-dried PHEMA gel (modified by PEG with MPEG 2000 chain length, reproduced with permission from [79]), (i) bioplotted PCL scaffold, (j) bioplotted PLLA scaffold, and (k) bioplotted gelatin scaffold and hydrogel.

**Figure 3:** (a) Microfluidic vessel networks: schematic cross-sectional view showing (i) morphology and barrier function of endothelium, (ii) endothelial sprouting, (iii) perivascular association, and (iv) blood perfusion, (b) schematic of microfluidic collagen scaffolds after fabrication, (c) *Z*-stack projection of horizontal confocal sections of endothelialized microfluidic vessels showing (i) overall network, (ii) views of corner, and (iii) branching sections (scale bar: 100 *μ*m ((a), (b), and (c) were reproduced with permission from [101]), (d) tube formation of autologous endothelial progenitor cells from adipose tissue in 3D scaffolds before and after labeling with lipophilic fluorochrome chloromethylbenzamido dialkylcarbocyanine showing the formed capillary-like structures in the Matrigel, (e–h) after seeding on BAM (cells, dual positive fluorescence, cell nucleus, and capillary-like structures are in red, yellow, blue, and green colors, respectively, scale bar = 100 *μ*m, reproduced with permission from [102]), (i–k) stereomicroscopic images of HOB-HDMEC spheroids indicated by arrows: (i) directly, (j) day 3, and (k) day 14 after transplantation (scale bars = 13 mm, reproduced with permission from [103]), (l) a vascular network after nine days in culture, a channel (optical thickness and z-position = 10 *μ*m) showing the endothelial monolayer lining the vascular lumen (scale bar = 200 *μ*m), and (m) endothelial cells formed single and multicellular sprouts from patterned vasculature, as shown in a *z*-stack (optical thickness = 200 *μ*m) from deeper within the gel (*z*-position = 300 *μ*m, left) ((l) and (m) were reproduced with permission from [22]).

**Figure 4:** Growth factor loading and release mechanism for tissue-engineered scaffolds: (a) direct approach, (b) loading mechanism in microspheres, and (c) GFs release by stimuli.

**Figure 5:** Vectors or transfected cells delivery approach in a scaffold for prolonged release of growth factors.

**Table 1:** Influence of biological factor on tissue vascularization.

Biological factor	Percentage/dosing amount	Scaffold details	Fabrication method	*In vitro/in vivo*	Results/findings	Reference
PLLA enriched with basement membrane proteins (Matrigel)	5% PLLA	6 × 6 × 1 mm	Solvent-casting particulate leaching	*In vivo*	Creation of uniform, branched microvascular network	[91]
Silk fibroin micronets	—	5 × 5 mm	3D nonwoven substrates made by boiling cocoons and soaking in 98% formic acid	*In vivo*	Promising vascularization by preculturing with osteoblasts	[157]
Gelatin-based sacrificial filament was embedded into a collagen scaffold	10% gelatin and 3.0 mg/mL collagen	Channels in the range of 0.7–1.5 mm for the width and 0.5–1.2 mm for the height	3D bioprinting	*In vitro* (human umbilical vein endothelial cells)	Supporting the viability of tissue up to 5 mm in distance at 5 million cells/mL density under the physiological flow condition	[1, 158]
Human outgrowth endothelial cells (OECs)	Starch-poly(caprolactone)	—	As described in [159]	*In vivo*	Osteoblasts played a pericyte‐like role and supported OEC-derived vessels	[159]
Fibroblast growth factor-loaded microspheres	Alginate scaffold (2% (w/v)) that incorporates tiny poly(lactic-co-glycolic acid) microspheres	High porosity (90%) with an average pore size of 130 microns	As described in [160]	*In vitro* basic fibroblast growth factor (bFGF)	The released bFGF induced the formation of large and matured blood vessels	[161]
Vascular endothelial growth factor (VEGF), platelet-derived growth factor-BB (PDGF-BB), and transforming growth factor-*β*1 (TGF-*β*1)	Alginate-sulfate/alginate (1% (w/v) solution of sodium alginate and a 0.3% (w/v) solution of hemicalcium gluconate for alginate crosslinking)	Diameter of 11 mm and thickness of 3 mm	Freeze-dry technique	*In vivo*	Creation of mature vessels after 3 months	[124]
VEGF and Ang-1	Hyaluronan (HA)	—	As described in [159]	*In vivo*	Creation of higher microvessel density after 14 days	[116]
FGF-4 plasmid	Gelatin hydrogel	—	Injection of GHG-DNA complex into the hindlimb muscle	*In vivo*	Promotion of angiogenesis in the newly developed tissues in the GHG-FGF4 group than the naked FGF4-gene four weeks after gene transfer	[147]
Plasmid encoding PDGF	Subcutaneously implanted PLG sponges	—	Gas foaming/particulate-leaching process	*In vivo*/*in vitro*	Improvement of ECM deposition and capillary formation	[148]
Plasmid-mediated VEGF	PLGA nanoparticles	—	Injection of the suspension of VEGF-loaded nanoparticles (VEGF-NPs) into myocardial tissues	*In vivo*	Higher capillary number compared to the naked plasmid DNA group	[149]
